The article "A Novel Triterpenoid Isolated from the Root Bark of Ailanthus excelsa Roxb (Tree of Heaven), AECHL-1 as a Potential Anti-Cancer Agent" was retracted in 2020. Reasons: lack of ethics approval or compliance; ethical violations by an author.

# A Novel Triterpenoid Isolated from the Root Bark of *Ailanthus excelsa* Roxb (Tree of Heaven), AECHL-1 as a Potential Anti-Cancer Agent

**DOI:** 10.1371/journal.pone.0005365

**Published:** 2009-04-28

**Authors:** Manish S. Lavhale, Santosh Kumar, Shri Hari Mishra, Sandhya L. Sitasawad

**Affiliations:** 1 Pharmacy Department, Faculty of Technology and Engineering, The M. S. University of Baroda, Vadodara, Gujarat, India; 2 National Centre for Cell Science, NCCS Complex, University of Pune Campus, Ganeshkhind, Pune, Maharashtra, India; Cleveland Clinic, United States of America

## Abstract

**Background:**

We report here the isolation and characterization of a new compound Ailanthus excelsa chloroform extract-1 (AECHL-1) (C_29_H_36_O_10_; molecular weight 543.8) from the root bark of *Ailanthus excelsa* Roxb. The compound possesses anti-cancer activity against a variety of cancer cell lines of different origin.

**Principal Findings:**

AECHL-1 treatment for 12 to 48 hr inhibited cell proliferation and induced death in B16F10, MDA-MB-231, MCF-7, and PC3 cells with minimum growth inhibition in normal HEK 293. The antitumor effect of AECHL-1 was comparable with that of the conventional antitumor drugs paclitaxel and cisplatin. AECHL-1-induced growth inhibition was associated with S/G_2_-M arrests in MDA-MB-231, MCF-7, and PC3 cells and a G_1_ arrest in B16F10 cells. We observed microtubule disruption in MCF-7 cells treated with AECHL-1 in vitro. Compared with control, subcutaneous injection of AECHL-1 to the sites of tumor of mouse melanoma B16F10 implanted in C57BL/6 mice and human breast cancer MCF-7 cells in athymic nude mice resulted in significant decrease in tumor volume. In B16F10 tumors, AECHL-1 at 50 µg/mouse/day dose for 15 days resulted in increased expression of tumor suppressor proteins P53/p21, reduction in the expression of the oncogene c-Myc, and downregulation of cyclin D1 and cdk4. Additionally, AECHL-1 treatment resulted in the phosphorylation of p53 at serine 15 in B16F10 tumors, which seems to exhibit p53-dependent growth inhibitory responses.

**Conclusions:**

The present data demonstrate the activity of a triterpenoid AECHL-1 which possess a broad spectrum of activity against cancer cells. We propose here that AECHL-1 is a futuristic anti-cancer drug whose therapeutic potential needs to be widely explored for chemotherapy against cancer.

## Introduction

According to the World Health Organization based on morbidity, mortality, economic burden, and emotional hardship, cancer may be considered the most onerous health problem afflicting people worldwide [1]. Currently, over 22.4 million people in the world are suffering from cancer. Approximately 10.1 million new cases are diagnosed with cancer annually, and more than 6.2 million die of the disease in the year 2000 [2]. This represents an increase of around 19% in incidence and 18% in mortality since 1990. An important aim of cancer research is to find therapeutic compounds having high specificity for cancerous cells/tumor and fewer side effects than the presently used cytostatic/cytotoxic agents.

Numerous plant-derived compounds used in cancer chemotherapy include vinblastine, vincristine, camptothecin derivatives, etoposide derived from epipodophyllotoxin, and paclitaxel (taxol®) [3]. However most of these compounds exhibit cell toxicity and can induce genotoxic, carcinogenic and teratogenic effects in non-tumor cells, and some of them failed in earlier clinical studies [4], [5]. Another most widely used metal-based drug at present against selected types of cancers is cisplatin [6], but use of cisplatin in curative therapy was associated with some serious clinical problems, such as severe normal tissue toxicity and resistance to the treatment [7]. These side effects limit their use as chemotherapeutic agents despite their high efficacy in treating target malignant cells. Consequently, new therapies and treatment strategies for this disease are necessary for treating patients with this disease. Therefore, the search for alternative drugs that are both effective in the treatment of cancers as well as non-toxic to normal tissue is an important research line [8].

Terpenoids are used extensively for their aromatic qualities. They play a role in traditional herbal remedies and are under investigation for antibacterial, antineoplastic, and other pharmaceutical functions. Natural triterpenoids, such as oleanolic acid and ursolic acid, are compounds with anti-tumorigenic and anti-inflammatory properties [9]. Synthetic triterpenoid derivatives such as 2-Cyano-3, 13 dioxooleana-1,9(11)-dien-28-oic acid (CDDO) [10] and its derivative 1-[2-cyano-3-,12-dioxooleana-1,9(11)-dien-28-oyl] imidazole (CDDO-Im) [11] also have anti-tumor activity. Root bark of *Ailanthus excelsa* Roxb (Tree of Heaven), a tree belonging to family *Simaroubaceae* is widely used in Ayurveda as evidenced by phytotherapy [12]. Other species from this family are well known for their anti-cancer activities [13]. Chemical constituents of *A. excelsa* include some triterpenes and alkaloids [14]. In the present study we have evaluated the *in vitro* and *in vivo* anti-cancer activity of a novel triterpenoid, AECHL-1 isolated from the root bark of the plant and found to be highly effective in cancer cells of different lineage.

## Materials and Methods

### Isolation and characterization of AECHL-1

The root bark of *A. excelsa* was botanically verified by Professor Shrihari Mishra (one of the authors in the present manuscript) and the extraction and fractionation of air-dried powdered root bark was done using chloroform. Isolation of AECHL-1 was done using silica gel column chromatography and characterized by ultra violet (Shimadzu 1700), infra red (Perkin Elmer Spectrum RX1), nuclear magnetic resonance (Bruker Avance I NMR Spectrometer) and mass spectroscopy (by Jeol SX 102 mass spectrometer). The purity of the AECHL-1 was assessed by HPLC on a RP C-18 Phenomenex column using methanol-water (90∶10, volume for volume) as the mobile phase. The purified compound, AECHL-1 was dissolved in DMSO as stock solutions.

### Cell lines

Normal human embryonic kidney cell line (HEK 293), mouse melanoma B16F10 cells (B16F10), human breast carcinoma (MDA-MB-231), human breast adeno-carcinoma (MCF-7) and human prostate (PC3) cells were obtained from ATCC (Manassas, VA). HEK 293, MCF-7 and B16F10 cells were cultured in Dulbecco's modified Eagle's medium and PC3 in Ham's F-12 media (Gibco) at 37°C under 5% CO_2_. MDA-MB-231 cells were cultured in Leibovitz's L-15 (Gibco) supplemented with 10% FCS (Gibco), 100 units/ml penicillin and 100 µg/ml streptomycin in a humidified atmosphere at 37°C.

### Cell viability assay

Direct interference between different concentrations of AECHL-1 (0–200 µM) and MTT in a cell-free system was not observed, therefore, MTT assay was used to test cell viability in the current system. HEK 293, B16F10, PC3, MCF 7 and MDA-MB-231 cells (4×10^3^/well) were cultured in 96-well plates and after 24 h treated with different concentrations of AECHL-1 (0–200 µM), cisplatin (0–100 µM) or paclitaxel (0–50 µM) for 12, 24, and 48 hr at 37°C. Cell viability was assessed by MTT (0.5 mg/ml) conversion as described previously [15].

### Cell proliferation assay

Proliferation of MCF-7 cells was determined by measuring (^3^H) thymidine incorporation. Briefly, aliquots of complete medium containing 4×10^3^ cells were distributed into 96-well tissue culture plates. After 24 hr, the media were replaced with various concentrations of the AECHL-1 (0–100 µM), cisplatin (0–100 µM) or paclitaxel (0–50 µM). Six hours after the treatment 1 µCi/well (^3^H) thymidine (Board of Radiation and Isotope Technology, Mumbai, India) was added and the cultures were incubated further for 42 hr at 37°C. Cells were rinsed and collected in scintillation mixture, and radioactivity incorporated into the DNA was determined with a liquid scintillation counter (Canberra Packard).

### Annexin V-FITC binding assay

B16F10, MDA-MB-231 and MCF-7 cells (3×10^5^/ml) were treated with various concentrations of AECHL-1 (0–40 µM) for 24 hr at 37°C. Cells were harvested after 24 hr, apoptosis was detected by using Annexin V-FITC apoptosis detection Kit (Calbiochem, USA) with flow cytometry (FACS Vantage–BD Sciences, USA). The data was analyzed using Cell Quest software for determining the percent of apoptotic cells.

### Cell cycle analysis

B16F10, PC3, MDA-MB-231 and MCF-7 cells (3×10^5^/ml) were treated with various concentrations of AECHL-1 (0–100 µM), or paclitaxel (0–10 µM) for 24 hr. Cell cycle analysis was performed as described earlier [16], with flow cytometry (FACS Vantage–BD Sciences, USA). The data was analyzed using Cell Quest software.

### Immunocytochemistry

MCF-7 cells were fixed with 3.7% paraformaldehyde, and then incubated with anti-α-tubulin antibodies (1∶10000; Sigma, St. Louis, MO). After the antibodies were washed off, the cells were incubated with alexa-conjugated secondary antibodies (1∶200; Sigma, St. Louis, MO). Images were captured with a confocal laser scanning microscope (Zeiss LSM510).

### Animal tumor models

Male C57BL/6 (6–8 weeks of age) and female athymic nude mice, NIH, nu/nu Swiss (10 weeks) were maintained in accordance with the Central Animal Ethical Committee procedures and guidelines. B16F10 melanoma cells were harvested, suspended in PBS, and subcutaneously injected into the right flank (2×10^6^ cells/flank) of C57BL/6 mice and MCF-7 cells (5×10^6^ cells/flank) into female athymic nude mice. Each athymic mouse was implanted subcutaneous with a 0.72-mg of 17-β-estradiol pellets, 2 weeks before inoculation of MCF-7 cells [17], [18]. Tumor size was measured every 3–4 days by a caliper and tumor volumes determined by the length (*L*) and the width (*W*): *V* = (*LW* ^2^)/2 [19]. After two weeks, AECHL-1 (50 µg), AECHL-1 (100 µg), cisplatin (100 µg) and PBS as vehicle control were injected subcutaneously to the site of tumor for 15 days in C57BL/6 mice (n = 6) and AECHL-1 (5 µg), AECHL-1 (10 µg), paclitaxel (20 µg) and PBS as vehicle control were injected subcutaneously to the site of tumor per day for 10 days in female athymic nude mice (n = 6). Tumor volume was measured at regular interval during the study. At the end of the experiment tumor and other organs were dissected out for histological analyses and western blots.

### Immunohistochemistry

Tissues and organs of C57BL/6 and nude mice were fixed in alcohol formalin for 24 hr and embedded in paraffin as previously described [20]. Tissue sections (5 µm) were stained with hematoxylin and eosin (H & E), visualized and photographed with an inverted microscope (Nikon, ECLIPSE, TE2000-U, Japan).

### Immunoblotting

Tumor tissue was homogenized in RIPA buffer (20 mM Tris–HCl pH 7.5, 120 mM NaCl, 1.0% Triton ×100, 0.1% SDS, 1% sodium deoxycholate, 10% glycerol, 1 mM EDTA and 1× protease inhibitor cocktail, Roche) proteins were isolated in solubilized form and concentrations were measured by Bradford assay (Bio-Rad protein assay kit). Solubilized protein (60 µg) was denatured in 2× SDS-PAGE sample buffer (sigma), resolved in 10% SDS–PAGE and transferred to nitrocellulose membrane followed by blocking of membrane with 5% nonfat milk powder (w/v) in TBST (10 mM Tris, 150 mM NaCl, 0.1% Tween 20). The membranes were incubated with rabbit polyclonal anti-p21 and anti-pp53 antibodies (1∶1000; Santa Cruz, CA), mouse monoclonal anti-CDK4, anti-Cyclin D1 antibodies (1∶1000; Cell Signaling Technology, Beverly, MA), mouse monoclonal anti-c-Myc antibody and mouse monoclonal anti-p53 antibody (1∶1000; Abcam, USA), followed by HRP-conjugated appropriate secondary antibodies and visualized by an enhanced chemiluminescence (Pierce) detection system. Membranes were stripped and re-probed with β-actin primary antibody (1∶10000; MP Biomedicals, Ohio, USA) as a protein loading control.

### Statistics

The data reported for tumor volumes are expressed as mean±SEM. Statistical differences were determined by ANOVA and post test applied was Tukey-Kramer multiple comparison Test.

## Results

### Chemistry: Ultraviolet, infra red, nuclear magnetic resonance, and mass characterization of AECHL-1

IR (KBr): 3425, 3419 (hydroxyl group), 2972, 2966, 2923, 2873 (alkyl C-H stretch), 1733 (δ lactone), 1718 (Bi acetyl), 1680 (C = O conjugation with alkene), 1652 (-C = C stretching), 1600 (aromatic), 1492, 1454, 1394 (methyl stretching), 1222 (δ lactone), 1184, 1110, 1051, 1031 (acetals), 1018 nm (alkanes). ^1^H-NMR (DMSO, 400 Hz) δ: 0.95 (3H, *t*, 4′-CH_3_), δ:1.15 (3H, d, H-24), δ:1.235 (3H, d, 5′-CH_3_), δ: 1.5 (2H, ddd, 5′-CH_2_), δ: 1.73 (3H, ddd, H-21), δ: 1.83 (1H, s, H-9), δ: 1.87 (1H, s, H-14), δ: 1.9 (2H, s, H-18), δ: 2.16 (3H, s, H-18), δ: 2.3 (3H, d, H-19) δ: 2.71 (2H, s, H-20), δ: 3.45 (2H, dd, H-23), δ:3.65 (2H, d, H-22), δ: 3.95 (1 H, t, H-12), δ: 4.05 (2H, s, H-22), δ: 5.30 (1H, s, H-15), δ: 5.46 (1H, s, OH-2), δ: 5.73 (1H, d,OH-2′), δ: 6.89 (1H, s, H-3), δ: 8.82 (1H, s, OH-11).

Fast atom bombardment mass spectroscopy: *m/z:* 1068 due to dimmer formation. The actual (M^+^) was considered to be 543.8, 463.3 (M-C_4_H_1_O_2_), 461.4 (M-C_4_H_2_O_2_), 459.4 (M-C_4_H_4_O_2_), 361.2 (M-C_9_H_11_O_4_) (Figure 1B) and Mass Spectra (Figure S1). AECHL-1 is a solid, mp. 248–250°C possessed a molecular formula of C_29_ H_36_O_10_ as indicated by EI and ES mass spectra. The IR spectrum showed the presence of hydroxyl (s) (3425 nm, 3419 nm), δ lactone (1733 nm), and aromatic moiety (1600 nm). The UV spectrum gave a characteristic absorption maximum at 235 nm, indicating the presence of auxochromic groups like hydroxyl and ketone. The ^1^H-NMR spectrum of AECHL-1 revealed the presence of an aromatic proton δ 6.89 and a singlet at δ 5.30 which is characteristic of the ester function at C-15. H-22 appeared as an AB system as a singlet at δ 4.05 and doublet at δ 3.65 and H-12 appeared as a triplet at δ 3.95. The methyl group H-19 on the aromatic ring appeared as singlet at δ 2.3. A doublet at δ 1.235 for six protons is assigned at H-5′. H-4′ appeared as a triplet at δ 0.95. The methyl group, H-18 appeared as a singlet at δ 2.16 (Figure 2).

**Figure 1:** Purity of AECHL-1 as assessed by HPLC. Single peak indicated that the preparation was >99% pure.

**Figure 2:** Structure of AECHL-1 with its mass fragments by NMR spectroscopy.

### Inhibition of cell viability, proliferation, and apoptosis by AECHL-1

Effect of AECHL-1 on the viability of B16F10, PC3, MDA-MB-231 and MCF-7 cells was assessed. AECHL-1 inhibited cell growth of MCF-7 cells in a concentration- and time-dependent manner by MTT assay (Figure 3A). AECHL-1 inhibited cell growth in different cancer cell lines with a minimum growth inhibition in HEK 293 at 48 hr (Figure 3B). HEK 293 treated with 200 µM AECHL-1 exhibited high survival rate (>90%) as compared to cancer cells. AECHL-1 was found to be more effective on MCF-7 in comparison with B16F10, PC3 and MDA-MB-231 in cell proliferation inhibition as observed by the (^3^H) thymidine uptake after 48 hr (Figure 3C). Moreover, AECHL-1 was found to be more potent than paclitaxel or cisplatin in cell proliferation inhibition in MCF-7 cells after 48 hr (Figure 3D).

**Figure 3:** Growth inhibition and cell proliferation of different tumor cell lines by AECHL-1 in vitro. (A) Cell growth by MTT assay in MCF-7 cells were treated with different concentrations of AECHL-1 (10, 20, 40 and 100 µM) for 12, 24 and 48 hr and cell viability was determined by MTT assay; (B) Cell growth by MTT assay in B16F10, PC3, MDA-MB-231 MCF-7 and HEK-293 cells. Cells were treated with different concentrations of AECHL-1 (10, 20, 40 100 and 200 µM) for 48 hr, and cell viability was determined by MTT assay; (C) Cell proliferation by (^3^H) thymidine incorporation in B16F10, PC3, MDA-MB-231, and MCF-7 cells. Cells were treated with different concentrations of AECHL-1 (10, 20, 40 and 100 µM) for 48 hr, and cell proliferation was determined by (^3^H) thymidine incorporation; (D) Comparison of AECHL-1 with other chemotherapeutic drugs. MCF-7 cells were treated with different concentrations (5, 10, 20, and 50 µM) of paclitaxel, cisplatin and AECHL-1 for 48 hr, and cell proliferation was determined by (^3^H) thymidine incorporation. Data are means±SEM of three independent experiments.

Annexin V-conjugated FITC and propidium iodide (PI) stain was used to analyze the total percentage of apoptotic cells induced by AECHL-1. The investigator to identify early apoptotic cells (Annexin V-FITC positive, PI negative), cells that are in late apoptosis (Annexin V-FITC and PI positive), the necrotic cells (PI positive only) and cells that are viable (Annexin V-FITC and PI negative). Total percentage of apoptotic cells increased up to 36.25% and 37.18% at 20 µM in B16F10, MDA-MB-231 cells respectively and 60.66% at 5 µM in MCF-7 cells (Figure 4).

**Figure 4:** Effect of AECHL-1 on apoptosis of tumor cells. Detection of apoptosis was done by the Annexin V-FITC apoptosis detection kit according to the manufacturer's instructions and then analyzed by flow cytometry: UR indicates the percentage of late apoptotic cells (Annexin V and PI positive cells), and LR indicates the percentage of early apoptotic cells (Annexin V positive cells) The data are presented in dot blots depicting annexin/fluorescein isothiocyanate (*x* axis) vs. PI staining (*y* axis). The percentage of cells in each quadrant is shown. The results are representative of three independent experiments.

### AECHL-1 induced cell cycle arrest in cancer cells

To determine the phase of the cell cycle at which AECHL-1 exerts its growth-inhibitory effect, exponentially growing B16F10, PC3, MDA-MB-231 and MCF-7 cells were treated with different concentrations of AECHL-1 for 24 hr and analyzed by flow cytometry (Table 1). We observed that B16F10 cells treated with AECHL-1 showed an increase in the population in G_1_ phase (52.18–72.08 %) with a concomitant decrease in the percentage of cells in S-G2/M phase (47.98–26.16%), suggesting a G_1_ arrest. In contrast, the number of PC3, MDA-MB-231 and MCF-7 cells in S-G2/M phase increased from 42.91% to 57.62%, 49.40% to 77.16% and 45.13% to 70.97% respectively in response to treatment with AECHL-1 and a decreased in G1 phase from 55.65% to 39.02%, 49.54% to 22.82%, 53.67% to 27.85% respectively suggesting a growth arrest in S-G2/M phase in PC3, MDA-MB-231 and MCF-7 cells. Paclitaxel treatment showed an increase in the population of MCF-7 cells in G2/M phase (29.30% to 72.55%) with a decrease in the percentage of cells in G1 phase (48.30% to 4.62%) suggesting a growth arrest in G2/M phase (Table 1). These results suggest that inhibition of cell cycle progression could be one of the molecular events associated with selective anti-cancer efficacy of AECHL-1 in cancer cells.

**Table 1:** Cell cycle analysis of AECHL-1–treated cells.

Cell line	Compound	Conc. (µM)	Phase of cell cycle (% of cells)			
			Sub G_0_	G_1_	S	G_2_/M
B16F10	AECHL-1	0	0.24	52.18	21.39	26.59
		10	0.39	56.55	20.46	23.02
		20	0.65	57.67	18.4	23.6
		40	2.05	72.08	11.43	14.73
		100	7.82	64.04	15.41	13.23
PC3	AECHL-1	0	1.44	55.65	15.21	27.7
		10	1.66	50.74	16.21	30.94
		20	1.79	48.96	13.99	34.99
		40	4.14	44.26	17.71	33.82
		100	3.36	39.02	20.25	37.37
MDA-231	AECHL-1	0	1.48	49.54	25.79	23.61
		10	1.03	43.03	24.06	32.21
		20	0.95	33.18	28.63	38.01
		40	0.54	26.66	28.12	45.15
		100	0.58	22.82	30.99	46.17
MCF-7	AECHL-1	0	1.64	53.67	19.03	26.1
		4	1.61	35.04	27.2	36.65
		10	1.99	27.85	34.19	36.78
		20	1.81	29.68	37.44	31.98
		40	2.55	36.26	32.5	29.42
MCF-7	Paclitaxel	0	3.17	48.3	20.42	29.3
		1	3.45	4.62	18.65	72.55
		2	5.21	7.41	22.89	63.71
		5	3.98	5.34	18.35	72.86
		10	3.47	4.86	18.96	69.36

Effect of AECHL-1 on cell cycle progression in B16F10, PC3, MDA-231, MCF-7 and paclitaxel in MCF-7 cells in 24 hr of treatment. Cell cycles were analyzed using propidium iodide. DNA content was analyzed using FACS to determine the cell cycle distribution.

### Effect of AECHL-1 on cellular microtubules

Microtubule staining in control and cells treated with AECHL-1 and paclitaxel, showed that both AECHL-1 and paclitaxel resulted in microtubule disruption with an increase in the density of cellular microtubules and formation of thick microtubule bundles surrounding the nucleus in comparison to the untreated control cells (Figure 5).

**Figure 5:** Effect of AECHL-1 on microtubules. MCF-7 cells were treated with the vehicle as a control, AECHL-1 (5 µM) and paclitaxel (5 µM) as a positive control for 24 h, and microtubules (red) were visualized by indirect immunofluorescence. DAPI was used to stain the cell nuclei (blue). Representative of 25–30 cells each in 3 separate experiments.

### Effect of AECHL-1 on primary tumor volume in allograft and xenograft

We also examined the effects of AECHL-1 on the in vivo growth of primary tumors. Our preliminary studies showed that, of the various doses of AECHL-1 (0.5 to 5 mg/kg) injected intraperitoneal in C57BL/6 mice, the maximum tolerated dose was a single dose of 0.5 mg/kg that showed no obvious sign of toxicity when observed for one month. On this basis, the dose that was chosen was 50 and 100 µg/kg/day (a dose that was 10–20% of this maximum tolerated dose). On day 18 significant increase in tumor volume in control group (p<0.001) and a regression in tumor volume was evident in mice treated with 50 µg AECHL-1 (44.303±5.20 % (p<0.001)) and with 100 µg AECHL-1 (51.014±1.27% (p<0.001)). Tumors treated with 100 µg cisplatin showed a reduction of tumor volume (93.13±0.539% (p<0.001)). However, AECHL-1 (50 µg) vs. AECHL-1 (100 µg) was found to be non Significant (P>0.05). On day 24 control, AECHL-1 (50 µg) and AECHL-1 (100 µg) treated mice showed further increase in tumor volume (p<0.001) but mice treated with cisplatin showed reduction in tumor volume (p<0.001). However, although cisplatin showed further reduction in tumor volume, the damage caused to other organs was more than that in the AECHL-1 (50 & 100 µg) treated group in C57BL/6 mice (Figure 6A and 6B).

**Figure 6:** Effect of AECHL-1 on primary tumor volume in allograft and xenograft. (A) Photographs of C57BL/6 mice showing 4-week-old allograft tumor growth by B16F10 cells; *below,* excised tumors with respective mice; (B) Tumor volume was determined at timed intervals as described in “Materials and Methods”. Tumor volume of experimental animals after treatment with 50, 100 µg AECHL-1 and 100 µg cisplatin was compared with the tumor volume of control animals; (C) Photographs of athymic nude mice showing 4-week-old xenograft tumor growth by MCF-7 cells; *below,* excised tumors with respective mice; (D) Tumor volume of experimental animals after treatment with 5, 10 µg AECHL-1 and 20 µg paclitaxel was compared with the tumor volume of control animals. Results represent the mean±SE of six starting animals in each group. Significant differences between ^*^Intra group at each time point are represented as: ^ns^ p>0.05, ^*^p<0.05, ^**^P<0.01, ^***^P<0.001 and ^#^Inter group at different doses are represented as ^ns^ P>0.05, ^#^<0.05, ^##^P<0.01, ^###^P<0.001.

Since the cytotoxic doses of AECHL-1 for MCF-7 cells in vitro were very low, the doses selected for tumor xenografts in female athymic nude mice injected with MCF-7 cells were 5 and 10 µg. These doses showed regression in tumor volume as: 35.72±0.05% for 5 µg (p<0.001) and 28.55±0.06% for 10 µg (p<0.001) whereas tumors treated with 20 µg paclitaxel showed a regression in tumor volume (14.19±0.32% (p<0.05)), which was less than the AECHL-1 treated group (Figure 6C and 6D).

### Effects of AECHL-1 treatment on tumor suppressor and cell cycle regulatory proteins in Tumor allograft of C57BL/6 Mice

We evaluated the effect of AECHL-1 treatment on the expression of the tumor suppressor protein p53, the cell cycle regulatory protein Cyclin D and cdk4 and the oncogene c-Myc. As shown in Figure 4E, AECHL-1 at 50 µg/mouse/day administered to B16F10-implanted tumors in C57BL/6 mice resulted in an increase in the expression of wild-type p53 protein and then decreased at a higher concentration (100 µg/mouse/day). The level of the p53 was greater in the AECHL-1-treated group than in the cisplatin-treated group, indicating that the antitumor action of AECHL-1 was different from cisplatin. Since phosphorylation at the Ser-15 residue of p53 is critical for p53-dependent activation of cell cycle regulatory proteins for G1 arrest, we determined the phosphorylation status of p53 and cyclin D1 and cdk4. AECHL-1 treatment resulted in an increase in phosphorylation of p53 at serine 15 residue in tumors at 50 µg/mouse/day with a concomitant increase in the level of p21 and decreased at 100 µg/mouse/day. Western blot analysis revealed that treatment with 50 and 100 µg/mouse/day AECHL-1 caused a significant reduction in the cycle-regulatory proteins cyclin D1 and cdk4. Treatment with 50 and 100 µg/mouse/day AECHL-1 also caused a significant reduction in the oncogene c-Myc thus indicating that inhibition of the cell cycle may be responsible for antitumor effects of AECHL-1 (Figure 7).

**Figure 7:** Effect of AECHL-1 on cell cycle regulatory proteins. Tumor tissue lysates were subjected to SDS-PAGE followed by Western immunoblotting. Membranes were probed with anti-p53, pp53, p21, c-myc, cyclin D1, cdk4, and β-actin antibodies followed by peroxidase-conjugated appropriate secondary antibodies, and visualized by enhanced chemiluminescence detection system. The experiments were repeated thrice with similar results and a representative blot is shown for each protein.

### Histological analysis of tumor tissue and other organs in C57BL/6 mice

Histological examination of tumor in C57BL/6 control mice showed well developed blood vessels, increased neovascularization, cell density and presence of hemorrhagic areas with probable signs of angiogenesis with increased possibility of metastasis (Figure 8.1A). Treatment of tumors with 50 µg AECHL-1 did not show much influence on the tumor vascularization but showed less occurrence of hemorrhagic areas, decrease in tumor cell density and occurrence of picnotic/necrotic cells in the center of the tumor (Figure 8.1B). Treatment with 100 µg AECHL-1 showed increase in necrotic cells, disappearance of neovascularization, hemorrhagic areas and low cell density compared to control (Figure 8.1C), thus indicating that AECHL-1 prevented the progression of angiogenesis and risk of metastasis by blocking neovascularization. Cisplatin treated group showed significant increase in necrotic cells, decrease in tumor cell density and volume (Figure 8.1D).

**Figure 8:** Histological analysis of tumor tissue and other organs in C57BL/6 and nude mice. (1) Representative H&E-stained sections from B16F10 allograft tumors and the characteristics of these tumors were analyzed (1A–1D). Morphological characteristics of heart (1E–1H), kidney (1I–1L), liver (1M–1P) and spleen (1Q–1T), six mice were used in each set of experiments. (2) Representative H&E-stained sections from MCF-7 xenograft tumors and the characteristics of these tumors were analyzed (2A–2D). Morphological characteristics of heart (2E–2H), kidney (2I–2L) and liver (2M–2P), spleen (2Q–2T), three mice were used in each set of experiments.

Compared with control, the heart tissue of the mice treated with 50 µg AECHL-1 showed normal structure while 100 µg showed extensive myocardial fiber necrosis and contraction bands. The fragmentation and smudging of the muscle fibers characteristic of coagulative necrosis was seen (Figure 8.1E–8.1G). Cisplatin treated mice also showed necrosis of myocardial fiber, slight lymphocytic infiltration and also fragmentation and smudging of the muscle fibers (Figure 8.1H).

Compared with control, the kidney of the mice treated with 50 µg AECHL-1 showed slight tubular vacuolization and tubular dilation with hemorrhagic areas with normal glomeruli appearing at the lower part. Treatment with 100 µg AECHL-1 showed tubular vacuolization, tubular dilation, hemorrhagic condition and scattered chronic inflammatory cell infiltrates (Figure 8.1I–8.1K). Cisplatin treated mice showed scattered lymphocytes in and around the vessel. Many neutrophils were also seen in the tubules and interstitium i.e. pyelonephritis (Figure 8.1L).

Compared with control, the liver of the mice treated with 50 µg AECHL-1 did not affect the normal architect. Mice treated with 100 µg AECHL-1 retained the normal architect of the liver (Figure 8.1M–8.1O). In cisplatin treated mice however, extensive necrosis of hepatocytes were seen. The arrow at the right side shows dead hepatocytes and this pattern can be seen with a variety of hepatotoxins, where focal hepatocytes necrosis with lymphocytic infiltration occurs. In these tissues, lesions look similar to that of Tyzzer's disease characterised by necrosis with varying degrees of inflammation in response to the necrosis. Acute hepatic lesions consist of necrotic foci surrounded by minimal, primarily neutrophilic, inflammation (Figure 8.1P).

Representative spleen sections from Control and mice treated with 50 µg AECHL-1 showed normal spleen architect and mice treated with 50 µg AECHL-1. Control and mice treated with 100 µg AECHL-1 and cisplatin showed hyperplasia of the white pulp, especially in the marginal zone (Ψ). Histology showed increased number of granulocytes in the marginal zones (Figure 8.1Q–8.1T).

### Histological examination of tumor tissue and other organs in nude mice

Tumors from control mice showed pronounced neovascularization throughout the section surrounded by highly dense cells and absence of necrotic cells (Figure 8.2A). AECHL-1 at 5 µg dose showed decreased tumor cell density and lacunae throughout the tumor area. It also showed loss of neovasulization and absence of hemorrhagic areas (Figure 8.2B). AECHL-1 at 10 µg showed many empty spaces, occurrence of hemorrhagic areas was seen but reduction in the vasculization was not seen (Figure 8.2C). Treatment with Paclitaxel lowered the tumor cell density with occurrence of many empty spaces and necrotic areas in the section (Figure 8.2D).

Treatment with 5 µg AECHL-1 did not show any change in the normal myocardium, while 10 µg AECHL-1 and Paclitaxel showed necrosis of myocardial fiber. Paclitaxel showed extensive myocardial fiber necrosis with fragmentation and smudging of the myocardium (Figure 8.2E–H). No significant change was observed in kidney structure from AECHL-1 treated groups, while paclitaxel treatment showed signs of tubular vacuolization dilation with hemorrhagic areas (Figure 8.2I–8.1L). Both AECHL-1 and Paclitaxel did not show any change in the normal architecture of liver (Figure 8.2M–8.2P) and Spleen sections (Figure 8.2Q–8.2T).

## Discussion

In the present study, we report a new anti-cancer compound AECHL-1, isolated from root bark of the plant *Ailanthus excelsa*. AECHL-1 was characterized by UV, IR, NMR and mass spectroscopy and the purity was conformed by HPLC. It is a triterpenoid with high polarity and a molecular weight 453.8 (Figure 1 and Figure 2). The tumor-suppressor gene p53 plays a vital role in the development of various types of cancers. It is estimated that 50% of all cancers develop due to mutations in p53 [21]–[23]. Therefore, we first tested the effect of AECHL-1 cytotoxicity and proliferation in four different cancerous cell lines with different tissue origin that contain either wild-type or mutant p53, as well as p53 null. B16F10 and MCF-7 cells contain wild type p53, MDA-MB-231 cells contain mutant p53 and PC3 cells are p53 null. Cisplatin, a highly DNA damaging agent and paclitaxel, a tubulin based anti-mitotic agent were used as positive controls.

We found that AECHL-1 inhibited the growth of MCF-7 cells in a concentration dependent manner at 12, 24 and 48 hr (Figure 3A). Cytotoxicity was also observed in the other cancer cells at 48 hr to a varying degree with a minimum growth inhibition of a normal human embryonic kidney cell line, HEK-293 (Figure 3B). The degree of cytotoxicity was MCF-7>B16F10>PC-3>MDA-MB-231>HEK-293 (Figure 3B) and inhibition of cell proliferation was MCF-7>B16F10>MDA-MB-231>PC-3 (Figure 3C).

Compared with paclitaxel and cisplatin, AECHL-1 showed greater potency in MCF-7 (Figure 3D), B16F10 and MDA-MB-231 cell proliferation inhibition at 24 and 48 hr (data not shown). These results indicate that in MCF-7, B16F10 and MDA-MB-231 cell line AECHL-1 is more effective in inhibition of cell proliferation than cisplatin or paclitaxel. However, in PC-3 cells, paclitaxel is more effective than cisplatin and AECHL-1.

In B16F10 cells, AECHL-1 was found to significantly induce cell cycle arrest in G1 phase, while in MCF-7, MDA-MB-231 and PC3 cells it showed arrest in S-G2/M phase in MCF-7 cells (Table 1).

The cell cycle arrest in AECHL-1 treated MCF-7 cells was followed by concentration dependent apoptosis, but the percentage of cell death was dependent on the types of cell lines. Compared to B16F10 and MDA-MB-231 cells, AECHL-1 was highly effective in MCF-7 cells at both high and low concentrations (Figure 4).

Therapeutic interference with the mitotic spindle apparatus is a widely used rationale for the treatment of tumors. The microtubule network required for mitosis and cell proliferation has been shown to be disrupted by the diterpenoid paclitaxel [24]. It has also been shown that microtubule disruption elevates p53 protein levels [25]. Our immunofluorescence staining of tubulin showed that similar to paclitaxel, AECHL-1 inhibited microtubule assembly (Figure 5).

Our in vitro results demonstrate that AECHL-1 can act as a new class of microtubule damaging agent arresting cell cycle progression at mitotic phase and inducing apoptosis. AECHL-1 was tested *in vivo* in C57BL/6 mice allograft with melanoma, B16F10 and nude mice xenograft with human breast cancer cells, MCF-7. Injections of AECHL-1 to the tumor sites were found to inhibit tumor growth in both models. In case of B16F10 melanoma model, a daily dose of 50 µg and 100 µg showed a significant antitumor effect, leading to regression of established tumors (Figure 6A and 6B) however; cisplatin was more effective than AECHL-1 but AECHL-1 showed less toxicity to kidney and heart while cisplatin showed greater damage to kidney, heart, liver and spleen (Figure 8.1). In the MCF-7 breast cancer model, a daily dose of 5 and 10 µg showed a significant antitumor effect, leading to regression of established tumors (Figure 6C and 6D).

In order to understand the major in vivo pathways through which AECHL-1 may induce tumor suppression, we studied the expression of the tumor suppressor, cell cycle regulatory proteins and oncogene in B16F10 melanoma. Our in vitro cell cycle analysis on B16F10 had showed a strong G1 arrest as a result of AECHL-1 treatment. Furthermore, mechanistic investigation in vivo in B16F10 tumor showed that both 50 µg of AECHL-1 and cisplatin up regulated the expression of p53 (Figure 7). However, AECHL-1 induced hyper phosphorylation of p53 at ser-15. Phosphorylation of p53 at ser15 help in strongly binding p53 to DNA for the up regulation of cell cycle regulatory proteins that helps in suppression of the growth of tumor [26]. Cisplatin also up regulated p53, but phosphorylation at ser-15 was not observed (Figure 7). This may be due to the fact that cisplatin suppress the growth of tumor cells by DNA damage and apoptosis [27]. The observation that ser-15 phosphorylation is required for p21 induction prompted us to investigate its role in G1 arrest [26], [28]. We found an increase in the expression of p21 in the AECHL-1 treated tumors. p21 forms a complex with CDK2/CDK4/CDK6 and inhibit the CDK-cyclin kinase activity phase [28], [29] and arrest the cells in G1 phase. c-Myc is an oncogene that is up regulated in cancer cells and help in the tumor growth [30]. We observed that treatment of AECHL-1 resulted in a marked decrease in c-Myc, CDK-4 and cyclin D1 levels that is known to arrest the cell in G1 [31]. Decreases level of c-Myc is known to be involved in the down regulation of cyclin D1 and CDK4 [32] (Figure 7). This also decreases the kinase activity and arrest the cell in G1 phase.

In conclusion, our data clearly show that AECHL-1 is less toxic, more selective, and more effective in the treatment of cancer in comparison to plant derived anti-cancer compound paclitaxel and metal-based compound cisplatin. It is efficacious in inhibiting the proliferation of a broad range of cancer cells as well as solid tumors. The novel compound AECHL-1 is found to interact directly with tubulin, arrest the cell cycle, and induce apoptosis of tumor cells. The antitumor effect of AECHL-1 was comparable with or even superior to the conventional chemotherapeutic drugs tested. The positive outcomes of such an in vitro and in vivo study could form a strong basis for the development of AECHL-1 as a novel agent for human cancer prevention and/or intervention.

## Supporting Information

Figure S1 (154 KB DOC)
